The article "Panax notoginseng Saponin Promotes Bone Regeneration in Distraction Osteogenesis via the TGF-β1 Signaling Pathway" was published in 2021. Journal: Evid Based Complement Alternat Med.

# *Panax notoginseng* Saponin Promotes Bone Regeneration in Distraction Osteogenesis via the TGF-*β*1 Signaling Pathway

**DOI:** 10.1155/2021/2895659

**Published:** 2021-10-21

**Authors:** Di Liu, Zhenchen Zhao, Weidong Jiang, Peiqi Zhu, Xiaoning An, Yu Xie, Xuanping Huang, Nuo Zhou

**Affiliations:** ^1^Department of Oral and Maxillofacial Surgery, Hospital of Stomatology, Guangxi Medical University, Nanning 530021, China; ^2^Guangxi Key Laboratory of Oral and Maxillofacial Rehabilitation and Reconstruction, Guangxi Key Laboratory of Oral and Maxillofacial Surgery Disease Treatment, Guangxi Clinical Research Center for Craniofacial Deformity, Nanning 530021, China

## Abstract

Distraction osteogenesis (DO) is an efficient strategy that is employed for the treatment of large bone defects in craniomaxillofacial surgery. Despite its utility, however, DO is associated with a prolonged consolidation phase and a high complication rate that hinder its more widespread utilization. *Panax notoginseng saponin* (PNS) is a traditional Chinese medicine that is frequently administered for the treatment of a range of conditions. Herein, we explored the ability of PNS treatment to influence osteogenic differentiation using both rabbit bone marrow mesenchymal cells (BMSCs) and a model of mandibular DO. BMSC proliferation was assessed via CCK-8 assay, while osteogenic differentiation was monitored through ALP and alizarin red S staining. A PCR approach was used to evaluate the expression of genes associated with osteogenesis (ALP, Runx2, and OCN) and genes linked to the TGF pathway (T*β*R-II, SMAD2, SMAD3, and PPM1A). For *in vivo* experiments, treated BMSCs were locally injected into the DO gap, with PNS being injected into treated rabbits every other day throughout the experimental period. The quality of the regenerative process was assessed *via* scanning electron microscopy (SEM), energy dispersive spectroscopy (EDS), X-ray imaging, and hematoxylin and eosin (H&E) staining. These analyses revealed that PNS was able to promote BMSC osteogenesis and mandibular generation, driving the upregulation of osteogenesis-related genes at the mRNA levels through the modulation of the TGF-*β*1/Smad pathway. Consistently, the overexpression or silencing of T*β*R-II in PNS-treated BMSCs was sufficient to modulate their osteogenic potential. Analyses of *in vivo* mandibular DO outcomes revealed significantly augmented new bone growth in the PNS-treated group relative to control animals, with maximal osteogenesis in the group overexpressing rabbit T*β*R-II. Together, these results highlight the PNS as a promising and cost-effective therapeutic tool with the potential to enhance bone regeneration in clinical contexts through the modulation of the TGF-*β*1/Smad pathway.

## 1. Introduction

Segmental mandibular bone defects arising as a consequence of skeletal abnormalities, tumor resection, or trauma can impair chewing functionality, result in undesirable facial aesthetics, and engender mental health problems that make the treatment of such defects an important clinical challenge in the field of oral and maxillofacial surgery [1]. Distraction osteogenesis (DO) has been shown to be an effective approach to repairing a range of craniofacial deformities [2]. Despite its benefits, however, DO necessitates a very prolonged treatment duration and is associated with a substantial risk of complications [3]. There is thus an urgent clinical need for the development of novel approaches to shortening the DO consolidation phase in clinical settings.

Stem cell-based therapeutic approaches have recently emerged as a promising approach to reducing DO-related complications by shortening the consolidation phase [4]. Mesenchymal stem cells (MSCs) are capable of undergoing self-renewal and differentiating into multiple cell types [5], and prior studies have explored their transplantation into damaged tissue sites in humans and animal models to facilitate tissue repair [6]. In the context of DO, MSCs can specifically migrate to the osteogenic front where they can undergo osteoblastic differentiation to facilitate new bone formation in response to mechanical tension [7]. Despite the clinical promise of MSC-based therapeutic strategies, however, the limited survival rates and inefficient differentiation of these cells following their transplantation limit their therapeutic utility [8].

*Panax notoginseng* saponin (PNS) is a traditional Chinese medicine composed of the primary bioactive components of *Panax notoginseng* (Sanqi), and it has been used to treat a range of conditions in China for centuries [9]. It has a long history of high clinical value, especially in promoting BMSC osteogenic differentiation [10] and angiogenesis [11]. However, the mechanisms whereby PNS may shape osteogenesis during DO remain to be defined. Herein, we sought to explore the pathways underlying PNS-mediated osteogenesis in an effort to provide a theoretical foundation for the therapeutic application of PNS as a tool to shorten the DO consolidation phase in clinical contexts.

## 2. Materials and Methods

### 2.1. Animal Surgery and DO Protocol

New Zealand white rabbits (3 months old; 2.5–3.0 kg) from the Experimental Animal Center of Guangxi Medical University (Nanning, China) were used for all experiments, which received approval from the Animal Care and Use Committee of Guangxi Medical University. In total, 14 rabbits were used for this study (Figure 1(a)). A 0.2% (v/v) xylazine and 2% pentobarbital sodium solution were administered to rabbits for anesthetization during surgery, after which all animals underwent a right mandibular osteotomy, with the osteotomy line being located between the mandibular first and second molars. The distal and proximal segments were then fixed using an internal distraction fixator (Zhongbang, China). Distraction was initiated following a 7-day latency phase (1 mm twice per day for 7 days) followed by a 0- or 14-day consolidation period whereafter pentobarbital sodium was administered to euthanize these animals (Figure 1(a)). Two of these rabbits developed infections prior to reaching the experimental endpoint and were thus excluded from the remainder of the study.

### 2.2. PNS and Lentivirus Therapy

To assess the therapeutic efficacy of PNS treatment in the context of DO-associated bone healing, these 14 experimental rabbits were randomly assigned to two groups that were administered 1 mL of either 120 mg/kg dose of PNS (*n* = 3) or 1 mL of saline (Ctrl, *n* = 3) daily after surgery. 1 × 10^6^ T*β*R-II overexpressing BMSCs were injected into the DO gap on the first day of the latency phase.

### 2.3. Digital Radiography

Immediately following distraction and after the consolidation period, X-ray (KAVO, USA) examinations were performed. Data were digitized using SIDEXIS XG 1.6 software, after which ImageJ software was used for densitometric measurements of the gray regions in the regenerating DO tissues in the right mandibular region of these experimental rabbits.

### 2.4. Hematoxylin and Eosin (H&E) Staining

After harvesting, tissues from the DO regeneration region were fixed for 48 h in 4% paraformaldehyde (PFA) at 4°C, after which they were treated for 4 weeks with 10% EDTA for decalcification. Samples were then paraffin-embedded, cut into 4 *μ*m sections using a rotary microtome (RM2255; Leica, Germany) along the long axis of each mandible in the sagittal plane, deparaffinized, and subjected to H&E staining to assess bone formation at the defect site.

### 2.5. Scanning Electron Microscopy

A 0.7 cm × 0.5 cm portion of the surface of the DO regeneration tissue region was excised, fixed using 3% glutaraldehyde, washed with PBS, dehydrated using an ethanol gradient, affixed to a sample table using a mixture of metal powder and low-resistance resin, and then sputter-coated with a metal coating solution under vacuum. Then, the tissue structure of each sample was assessed via scanning electron microscopy (SEM), with images being recorded.

### 2.6. BMSC Isolation, Culture, and Characterization

A density gradient centrifugation approach was used to collect mononuclear cells from the rabbit bone marrow with the Percoll cell separation solution (Solarbio, China), after which these cells were cultured in T25 cell culture flasks containing *α*MEM supplemented with 10% fetal bovine serum (FBS; Gibco, USA) and 1% penicillin-streptomycin (Gibco, USA) at 37°C in a humidified 5% CO_2_ incubator. Media were changed every 3 days, and rBMSCs from passages 3–5 were used for all experiments. The surface phenotype of these rBMSCs was assessed via flow cytometry by staining 5 × 10^5^ BMSCs from passage 3 with antibodies specific for CD34 (1 : 1000; BioLegend, CA, USA), CD45 (1 : 1000; BioLegend), CD90 (1 : 500; BioLegend), CD105 (1 : 1000; BioLegend), HLA-DR (1 : 1,000; Abcam, Cambridge, UK), and CD44 (1 : 1,000; Abcam) for 30 minutes at 4°C while protected from light. Cells were then rinsed with PBS and analyzed using a FACScan flow cytometry system (CytoFLEX; Beckman Coulter, USA).

### 2.7. Osteogenic Differentiation

BMSCs were seeded in 12-well plates (5000 cells/cm^2^) and allowed to grow until 80% confluent, at which time media were exchanged for osteogenic induction media (Sigma-Aldrich, MO, USA), PNS, and/or *α*-MEM, as appropriate. Following a 2-week induction period, cells were fixed using 4% PFA and stained using 2% alizarin red S (pH 4.2) and alkaline phosphatase (ALP).

### 2.8. Cell Transfection

T*β*R-II specific shRNA and overexpression lentiviral vectors (GeneChem, China) were transduced into cells at an MOI of 50 based on provided protocols. The siRNAs targeting the rabbit T*β*R-II gene (1#, 5′-GCAATGACCACATCATCTT-3′; 2#, 5′-CCTGGAATCCAGGATGAAT-3′; 3#, 5′-GGAGAAGATTCCAGAAGAA-3′) were used to specifically downregulate the level of T*β*R-II in BMSCs. For overexpression constructs, the full-length T*β*R-II (NM_001177748.1) sequence was cloned into the Ubi-MCS-3FLAG-SV40-EGFP-IRES-puromycin lentiviral vector prior to BMSC transduction, with control cells instead being transduced with a negative control (NC) lentivirus. At 48 h post-shRNA transfection, cells were collected to confirm knockdown efficiency via qPCR.

### 2.9. Quantitative Real-Time PCR (qRT-PCR)

Osteogenic-related and TGF-*β*1/Smad signaling pathway-related gene expressions were assessed on days 3, 6, and 12 of the osteogenic induction periods via qPCR. Briefly, cellular RNA was collected using TRIzol (Invitrogen, CA, USA) based on provided directions, and cDNA was prepared using a reverse transcription kit (Invitrogen). A QuantStudio-5 system (Applied Biosystems, USA) was then utilized for all qPCR amplification using the primers shown in Table 1. Relative gene expression was assessed via the 2^−ΔΔCT^ method, with GAPDH being used for normalization.

### 2.10. Statistical Analysis

SPSS 23.0 was used for all data analysis. Data are given as means with the standard deviation (SD) and were analyzed using Student's *t*-tests and ANOVAs after a Kolmogorov–Smirnov test was used to assess whether data conformed to a normal distribution. *p* < 0.05 was the significance threshold.

## 3. Results

### 3.1. PNS Administration Promotes Enhanced DO Regeneration

We found that callus formation was evident in the distraction gap in the context of DO immediately following the distraction phase in both the saline and PNS-treated rabbit groups in this study. More mineralized callus formation was evident in the PNS group relative to the control group at the DO14 and DO28 time points, however (Figures 1(a)–1(c)). Average DO callus bone density was measured through X-ray imaging (Figures 1(d) and 1(e)), which indicated a significant increase in bone density in the PNS group relative to the Ctrl group (*p* < 0.01) (Figures 1(f) and 1(g)). H&E staining further revealed that the distraction gap region in rabbits from the saline treatment group was largely filled with fibrous tissue, whereas in the PNS treatment group, this region was bridged by newly formed immature bone trabecula (Figures 1(h) and 1(i)). SEM imaging additionally revealed increased trabecular tightness following PNS treatment (Figures 1(j) and 1(k)). Together, these data suggested that PNS treatment can enhance bone regeneration *in vivo,* prompting us to conduct additional *in vitro* analyses aimed at understanding the mechanistic basis for this effect.

### 3.2. BMSC Isolation and Characterization

To begin exploring phenotypes pertaining to *in vitro* osteogenesis, BMSCs were isolated from the rabbit bone marrow via density gradient centrifugation. On day 3 of culture, a small number of adherent cells with irregular spindle-, polygon-, or star-like morphological conformations were observed (Figure 2(a)). On day 5 after seeding, colonies were evident (Figure 2(b)), and by day 8, these colonies had fused, exhibiting a swirl-shaped morphological conformation (Figure 2(c)). Then, the surface phenotypes of these putative rabbit BMSCs were assessed via flow cytometry, revealing them to be positive for MSC markers including CD44, CD90, and CD105, whereas they did not express the hematopoietic lineage markers HLA-DR, CD34, or CD45 (Figure 2(d)). When cultured in osteogenic media, these BMSCs promoted mineralized ECM formation as evidence by positive alizarin red S staining (Figure 2(e)).

### 3.3. PNS Treatment Enhances rBMSC Osteogenic Differentiation

Next, a CCK-8 assay approach was used to assess the proliferation of BMSCs cultured for 14 days in *α*-MEM supplemented with 100 mg/mL PNS (Figure 3(a)). Such treatment had no apparent impact on BMSC proliferation relative to control treatment, suggesting that PNS does not induce cytotoxicity in this assay context. Consistently, PNS treatment resulted in significant increases in the expression of osteogenic genes including *OCN*, *ALP*, and *Runx2* at the mRNA level (Figure 3(b)). Moreover, ALP (Figure 3(d)) and ARS (Figure 3(e)) were conducted, respectively, on day 7 and 14 of osteogenic induction, revealing relatively weak staining in the control group, whereas this staining was more pronounced for BMSCs that had been treated with PNS.

### 3.4. PNS Promotes BMSC Osteogenesis via the TGF-*β*1 Signaling Pathway

The TGF-*β*1/Smad signaling pathway plays a central role in regulating a variety of processes pertaining to cellular differentiation and proliferation in the context of wound healing and pathological settings [12]. To better understand how PNS treatment shapes BMSC osteogenesis, we, therefore, explored TGF-*β*1/Smad signaling pathway-related gene expression in these cells. This analysis revealed that BMSCs treated with PNS exhibited the pronounced upregulation of T*β*R-II, SMAD2, SMAD3, and PPM1A relative to control BMSCs at the mRNA and protein levels (Figures 3(b) and 3(c)). Together, these findings were suggestive of a role for the TGF-*β*1/Smad signaling pathway in the context of PNS-mediated osteogenesis.

To directly explore the importance of the TGF-*β*1/Smad signaling pathway in our models of PNS-mediated osteogenic regeneration, we next either overexpressed or silenced the TGF-*β* receptor T*β*R-II in BMSCs, confirming successful knockdown or overexpression via qPCR (Figure 4(a)). From a mechanistic perspective, the expressions of T*β*R-II, SMAD2, and SMAD3 were upregulated when T*β*R-II was overexpressed (Figure 4(b)), and T*β*R-II knockdown attenuated the PNS-mediated overexpression of these genes (Figure 4(c)). Moreover, the level of PPM1A was decreased in the OE group and enhanced in T*β*R-II deficiency BMSCs (Figures 4(b) and 4(c)). Western blot results further revealed that T*β*R-II overexpression was associated with higher phosphorylation levels of SMAD2 and SMAD3, while METTL3 knockdown reduced the levels of these key signaling proteins (Figure 4(d)). ALP and ARS were then used to assess BMSC osteogenic differentiation in the context of PNS treatment and T*β*R-II knockdown or overexpression. When this receptor was overexpressed, a significant increase in the ALP (Figure 4(e)) and the number of calcium nodes (Figure 4(f)) was evident in samples from cells treated with PNS, whereas T*β*R-II knockdown failed to exhibit an enhanced ALP activity (Figure 4(e)) and associated with only sporadic calcium nodule formation (Figure 4(f)) at a rate lower than that observed in the PNS treatment group. These findings thus suggested that BMSC osteogenesis was enhanced by PNS treatment in a manner dependent on the TGF-*β*1/Smad signaling pathway.

### 3.5. T*β*R-II Overexpression Accelerates *In Vivo* DO-Related Ossification

To more fully explore the role of T*β*R-II as a regulator of DO-mediated bone regeneration, 1 × 10^6^ BMSCs overexpressing T*β*R-II were injected into the DO gap at the start of the distraction period. Clear differences in overall local bone formation were evident in these different treatment groups, with maximal bone growth in the distraction gap being evident in the T*β*R-II overexpression group (Figures 5(a) and 5(b)). Both in 0-week (DO14) and 2-week consolidation period (DO28), higher callus bone density was evident in the T*β*R-II overexpression group (Figures 5(c)–5(f)). H&E staining indicated more robust trabecular formation in the DO gap in these groups (Figures 5(g)-5(h)), and SEM imaging yielded comparable results (Figures 5(i)-5(j)). When calcium and phosphorus levels were assessed via electron spectrometry, the ratio of calcium to phosphorus was also found to be higher in this T*β*R-II overexpression group relative to other groups (Figures 5(i)-5(j)).

## 4. Discussion

Despite being effective, the DO procedure necessitates a prolonged consolidation phase that can result in high complication rates [13], restricting its widespread clinical implementation. A range of factors has been explored as potential adjuvant therapies capable of improving DO-related bone regeneration, including growth factors [14], laser therapy [15], hormone [16, 17], bisphosphonates [18], and stem cell therapy [4]. While many of these approaches have been found to accelerate bone regeneration to varying extents, there are concerns regarding their safety or feasibility, which have limited their clinical use [19, 20]. Traditional Chinese medicines, in contrast, are orally administered compounds that are generally regarded as safe and are rarely associated with adverse side effects. While a few prior studies have found that PNS can be applied to enhance DO [21] and to promote angiogenesis [11], the mechanisms whereby this traditional medicinal preparation influences BMSC osteogenesis in the context of DO remains to be clarified. The present study was thus formulated to explore these mechanisms *in vitro* and *in vivo.*

We chose a PNS dose of 100 mg/mL for use in the present study, as our prior study indicated that this was an optimal therapeutic dose [22]. This study is the first to our knowledge to have explored the ability of PNS to modulate rBMSC proliferation and osteogenic differentiation or to explore the underlying mechanisms. We found that PNS was able to enhance osteogenesis and to promote the upregulation of genes associated with the osteogenic and TGF-*β* signaling pathways in rBMSCs. Runx2 is a transcription factor that serves as a master regulator of osteoblastic differentiation [23], which is essential for bone regeneration [24]. In these experiments, PNS treatment resulted in Runx2 and ALP upregulation in rBMSCs, which has the potential to favor osteogenesis during DO [25]. These findings thus suggest that PNS can promote BMSC osteogenesis while simultaneously enhancing osteogenic cytokine expression, which is a prerequisite for DO.

Isoforms of TGF-*β* and its receptors can influence the bone regeneration processes [26], favoring osteoblast differentiation while suppressing the activation of osteoclasts [27]. The activation of SMAD family proteins may promote rBMSC migration to the site of callus formation such that they can participate in bone healing [5]. Given the importance of the TGF-*β* signaling pathway in this regenerative context, we hypothesized that PNS exerts its pro-regenerative activity in a manner dependent on this pathway. PNS may promote the expression of TGF-*β*1 in rBMSCs, thereby promoting the upregulation of the TGF-*β*R2 membrane receptor and enhancing intracellular levels of SMAD2 and SMAD3, which can facilitate TGF*β*1 signal transduction. Under normal physiological conditions, PPM1A dephosphorylates SMAD2 and SMAD3, which are exported from the nucleus, thereby terminating TGF-*β* signaling [28, 29]. Nuclear PPM1A translocation was reduced in response to PNS stimulation in this study, indicating that PNS treatment was sufficient to inhibit PPM1A, thereby enhancing TGF-*β*1/Smad signal transduction to further promote BMSC osteogenic differentiation and function. However, further research will be needed to establish whether other pathways upstream or downstream of the TGF-*β* signaling pathway are also involved in migration, differentiation, and proliferation in the context of DO-mediated bone regeneration.

PNS has previously been purported to exhibit pro-bone metabolism, neuroprotective, hepatoprotective, renoprotective, antitumor, cardioprotective, antidiabetic, and other beneficial effects, in addition to being safe and convenient to use [30]. Prior evidence also suggests that PNS and its main bioactive component, NGR1, can stimulate the proliferation, differentiation, and mineralization of osteoblasts through the enhancement of cellular ALP activity, ECM mineralization, and osteoblast-associated gene expression [31, 32]. The results of the present study further confirmed that PNS administration was sufficient to enhance osteogenesis in a rabbit model of DO, with reductions in PPM1A expression together with the upregulation of TGF-*β*1/Smad signaling pathway genes (T*β*R-II, SMAD2/3), potentially favoring osteogenic differentiation and DO regeneration. Together, these findings confirm the ability of PNS to efficiently promote *in vivo* DO callus regeneration.

Herein, we determined that PNS was able to promote accelerated bone remodeling in the context of DO through a mechanism dependent upon the TGF-*β*1/Smad pathway, suggesting that PNS can be applied in clinical settings to improve DO-related treatment outcomes. In light of these findings, we plan to perform a prospective randomized controlled trial aimed at more fully exploring the impact of PNS injection on DO-related regeneration and angiogenesis. Our *in vitro* data revealed that PNS was able to directly enhance rBMSC osteogenesis through the enhancement of osteogenic differentiation and the upregulation of key osteogenesis-related genes. Such stimulation was linked to T*β*R-II activation and the suppression of PPM1A, highlighting a novel mechanism whereby PNS can be leveraged to accelerate DO-related bone regeneration. However, there are certain limitations to this study. For one, these results are derived from a rabbit model of DO, and further studies of larger animals such as dogs or pigs will be essential preclinical steps to better understand the therapeutic value of PNS in this regenerative setting, as these larger animals exhibit bone architecture more similar to that found in humans. Second, we only assessed bone regeneration over a two-week period, and future studies assessing consolidation over a four-to-six-week period will thus be important to more fully elucidate the value of PNS as a regenerative pharmaceutical compound. Third, although the TGF-*β*1/Smad signaling pathway plays an important role in osteogenesis, we did not consider other signaling pathways that play a role in osteogenesis. As such, future studies will need to employ RNA-seq approaches to fully elucidate the detailed mechanism underlying the ability of PNS. These will help us to further understand the role of PNS to accelerate the translation of PNS-related biological therapies into clinical practice.

## 5. Conclusion

In summary, our results indicate that PNS treatment can promote the osteogenic differentiation of rabbit BMSCs through the activation of the TGF-*β*1/Smad pathway *in vitro* and can accelerate mandibular regeneration in the context of DO *in vivo.* These findings provide new insights into the mechanisms whereby PNS can influence osteogenesis and offer a robust foundation for future studies seeking to explore the potential clinical utility of this traditional medicinal compound.

## Figures and Tables

**Figure 1:** PNS promotes the regeneration context of DO. (a) Rabbit model of DO. At the end of the distraction phase (DO14) and 2 weeks of consolidation (DO28), callus samples from the distraction gap were harvested for further study. (b, c) Mandible specimens for Ctrl and PNS-treated groups on day 14 (b) and day 28 (c) after surgery. The distraction gap featured more new bone tissue in the PNS group both on DO14 and DO28. (d, e) Images of radiograph. (f, g) The gray value of X-ray. (h, i) Histomorphologic results on DO14 and DO28. Compared with the control group, the distraction gaps of the PNS group showed increased fibrous and cartilaginous tissues in DO14. In DO28, numerous trabecular bones in the center zone occurred in the PNS group. (j, k) The SEM results of Ctrl and PNS-treated groups. Analyses were conducted using data from three independent experiments. ^*∗∗∗*^*p* < 0.001.

**Figure 2:** BMSC cultivation and identification. (a–c) The morphology of BMSCs at day 3 (a), day 5 (b), and day 8 (c) of culture. Cells displayed a typical elongated spindle shape. (d) Cell surface markers of BMSCs. Over 93% MSCs expressed the positive markers CD44, CD90, and CD105, while only a few cells (<1.2%) expressed the negative markers CD34, CD45, and HLA-DR. (e) The results of osteogenic induction were seen on alizarin red staining.

**Figure 3:** PNS promotes osteogenic differentiation of BMSCs. (a) CCK-8 assay for BMSCs cultured in 100 mg/mL concentrations of PNS at day 1 to 2 weeks. (b) Expressions of osteogenic-specific genes and TGF-*β*1/SMAD signaling pathway-related genes of BMSCs treated with PNS were assessed with qRT-PCR. (c) Western blot of SMAD2, p-SMAD2, SMAD3, p-SMAD3, and PPM1A in BMSCs treated with PNS. (d, e) Osteogenic differentiation of BMSCs treated with PNS was determined with ALP staining, ALP activity assay (d), and alizarin red staining (e). Data are means ± SD. ^*∗*^*p* < 0.05, ^*∗∗*^*p* < 0.01, and ^*∗∗∗*^*p* < 0.001.

**Figure 4:** PNS regulates osteogenic differentiation of BMSCs via the TGF-*β*1/SMAD signaling pathway. (a) Overexpression and inhibition of T*β*R-II were confirmed via qRT-PCR. (b, c) Following T*β*R-II knockdown or overexpression, the mRNA levels of the pathway-related genes were significantly altered. (d) WB analysis for the expression levels of SMAD2, p-SMAD2, SMAD3, p-SMAD3, and PPM1A treated with lentivirus. (e, f) T*β*R-II overexpression enhanced osteogenic differentiation, while silencing impairs such capability. (e) ALP staining and ALP activity assay. (f) Alizarin red staining. OE-NC and T*β*R-II-OE groups or NC-shRNA and T*β*R-II-inhibitor groups were compared *via* Student's *t*-tests. Data are means ± SD. ^*∗∗*^*p* < 0.01 and ^*∗∗∗*^*p* < 0.001.

**Figure 5:** T*β*R-II accelerated mature callus formation during distraction osteogenesis. (a–f) The gross observation (a, b) and X-ray (c–f) results showed that T*β*R-II could increase callus regeneration. (g, h) H&E staining showed that T*β*R-II was able to accelerate new bone formation. SEM (i, j) results from control and T*β*R-II groups revealed that the amount of mineralized callus increased both in DO14 and DO28. OE-NC and OE-T*β*R-II groups were compared *via* Student's *t*-tests. Data are means ± SD. ^*∗∗∗*^*p* < 0.001.

**Table 1:** Primer sequences.

Gene	Forward (5′-3′)	Reverse (5′-3′)
*Runx2*	CCGAAATGCCTCTGCTGTT	ACTCTTGCCTCGTCCACTCC
*ALP*	GCACAGCCACAGCCTACCT	CACGGACTTCCCTGCCTTC
*OCN*	TGATGCAAGCCTGACCTCC	CCATAGCCCACGGCCAAAA
*TβR-II*	TGGAGGAAGAACGATGAAAACA	ATGATACACTTTGGAGAGGCAGAA
*SMAD2*	CCATCTTGCCGTTCACTCC	CCTTCTCACACCACTTCTCTTCC
*SMAD3*	CAGCCACTCAACCACCCTTC	AAACGCCACACTCCAACTCAC
*PPM1A*	TTTCACCCCAGCACACTTACTTC	GATACAGCCAGAGAGCCATTCAC
*GAPDH*	CCACTTTGTGAAGCTCATTTCCT	TCGTCCTCCTCTGGTGCTCT

## Data Availability

The data used to support the findings of this study are included within the article.
